# Impact of vascular endothelial growth factor (VEGF) and vascular endothelial growth factor receptor (VEGFR) single nucleotide polymorphisms on outcome in gastroenteropancreatic neuroendocrine neoplasms

**DOI:** 10.1371/journal.pone.0197035

**Published:** 2018-05-22

**Authors:** Rossana Berardi, Mariangela Torniai, Stefano Partelli, Corrado Rubini, Silvia Pagliaretta, Agnese Savini, Vanessa Polenta, Matteo Santoni, Riccardo Giampieri, Sofia Onorati, Federica Barucca, Alberto Murrone, Francesca Bianchi, Massimo Falconi

**Affiliations:** 1 Clinica di Oncologia Medica, Università Politecnica delle Marche, Azienda Ospedaliero-Universitaria Ospedali Riuniti di Ancona, Ancona, Italy; 2 Chirurgia del Pancreas, Ospedale San Raffaele IRCCS, Università Vita e Salute, Milano, Italy; 3 Section of Pathological Anatomy and Histopathology, Deparment of Neuroscience, Università Politecnica delle Marche, Azienda Ospedaliero-Universitaria Ospedali Riuniti di Ancona, Ancona, Italy; 4 Dipartimento di Chirurgia Generale, Azienda Ospedaliero-Universitaria Ospedali Riuniti di Ancona, Ancona, Italy; Southern Illinois University School of Medicine, UNITED STATES

## Abstract

Angiogenesis represents a key event in cancer development, leading to local invasion e metastatization, and might be considered a basic feature in gastroenteropancreatic neuroendocrine neoplasms (GEP-NENs) with a high expression of angiogenic molecules. We aimed to analyze the prognostic and predictive role of angiogenic factors in GEP-NENs through the analysis of single nucleotide polymorphisms (SNPs) of VEGF-A, VEGFR2 and VEGFR3. The genomic DNA of 58 consecutive patients with GEP-NENs treated at our Institution was extracted from peripheral blood. Two SNPs were identified respectively in VEGF-A (rs2010963G>C, rs699947A>C), VEGFR-2 (rs2305948C>T, rs1870377T>A), and VEGFR-3 (rs307821T>C, rs307826C>A) gene. Gene polymorphisms were determined by Real-Time PCR using TaqMan assays. Median age was 57 years (range 24–79 years); 32 patients were male and 77.5% of NENs were localized in the pancreas. The allele frequency of VEGFR-2 rs2305948T and of VEGF-A rs2010963C showed a trend of higher frequency than in general population (12.1% vs. 8.0% and 34.5% vs. 31.2%, respectively). Three out SNPs (VEGF-A rs699947C, VEGF-A rs2010963GC and VEGFR-3 rs307821C) showed a correlation with an increased risk of disease relapse. Moreover median PFS changes according to the presence of 0–1 SNPs (20.7% of cases; 61.9 months), 2 SNPs (25.9%; 49.2 months) and 3 SNPs (53.4%; 27.8 months) (*p* = 0.034). Results suggest, for the first time, that specific SNPs in VEGF-A and VEGFR-3 correlate with poor prognosis in GEP-NENs. The identification of this new prognostic factor might be helpful in order to optimize the management of these heterogeneous neoplasms.

## Introduction

Gastroenteropancreatic neuroendocrine neoplasms (GEP-NENs) represent a heterogeneous family of diseases arising from homonym cells distributed in pancreatic islets and in the digestive tract.

The incidence of GEP-NENs has substantially increased 3.65-fold in the USA and 3.8 to 4.8-fold in Europe over the past four decades [1], primarily due to a considerable improvement of diagnostic tools.

Although traditionally considered slow progressing tumors, their clinical behaviour might be very aggressive [2] depending on tumor grading, disease staging and primary tumor site [3]. Moreover gender, race and year of diagnosis might affect overall survival rates [4].

Moreover, clinical management of GEP-NENs is still challenging and should be conducted under a multidisciplinary approach. Surgery still remains the only potentially curative therapeutic option, mainly depending on tumor size and patient’s performance status [5]. In locally-advanced and metastatic setting, medical therapy includes somatostatin analogues (SSAs), peptide receptor radionuclide therapy (PRRT), targeted agents as angiogenesis and mTOR (mammalian target of rapamycin) inhibitors and chemotherapy, but the optimal sequence still represents matter of debate [6].

Angiogenesis represents a key event in cancer development, delivering oxygen and nutrients to growing cells, and tumor progression, leading to local invasion e metastatization [7]. VEGF (Vascular Endotelial Growth Factor), also known as VEGF-A, belongs to a larger family of proteins [8] and represents the principal mediator of pathological angiogenesis [9]. VEGFs promote angiogenesis binding three main subtypes of tyrosine kinase receptors: VEGFR-1 (also known as FLT1), VEGFR-2 (FLK1) and VEGFR-3 (FLT4) [10]. Hypoxia secondary to tumor proliferation represents a major driver of VEGF production through the activation of HIF (Hypoxia Inducible Factor) pathway in tumor cells and in microenvironment [10]. Positive regulators of angiogenesis also include several mediators such as PDGF (platelet-derived growth factor), TGF (transforming growth factor) and EGF (epidermal growth factor) through a dysregulation in their production or a constitutive activation of their specific signalling pathways [11]. The genetic variability of these genes translating throught single nucleotide polymorphisms (SNPs) have been reported contributing to high variability in VEGF-A expression [12, 13].

Even VEGFs pathway has been extensively studied in order to identify new potential targets in the treatment of neuroendocrine neoplasms, the prognostic role of VEGFs and/or VEGFRs expression has not yet been clarified with conflicting results in the literature. In fact several studies seem to attribute a negative prognostic value to VEGFs/VEGFRs overexpression [14–16], while other studies challenge this hypothesis [17, 18].

On the basis of biological and clinical heterogeneity of GEP-NENs, patients’ stratification according to biomolecular characteristics seems necessary in order to better understand the role of antiangiogenic drugs optimizing their efficacy in specific subsets of patients.

On this scenario, we aimed to analyze the prognostic and predictive role of angiogenic factors in GEP-NENs through the analysis of SNPs (Single Nucleotide Polymorphisms). In particular, we evaluated the expression of some SNPs of VEGF-A, VEGFR-2 and VEGFR-3 focusing on their potential role in neoplasm susceptibly and their prognostic significance.

## Patients and methods

### Study population and data collection

The study population included all consecutive patients aged 18 years or older with histologically or cytologically proven diagnosis of GEP-NENs treated at our Institution from January 2004 to January 2016.

Recorded data were retrospectively collected from patients electronic medical records and paper charts and included gender, age, tumor grading (according to WHO 2010 classification [19]) and histological features, disease staging at the time of the diagnosis (according to the TNM Seventh edition (2010) [20]) and data regarding all the treatments received by the patients. All data were fully anonymized before we accessed them. All the patients had provided informed consent to have data from their medical records used in the research.

This study was carried out in accordance with the approval by the Ethical Committee of our Institution CERM (Comitato Etico Regionale Marche) and written informed consent for the biological procedures was obtained from each patient.

### SNPs selection, DNA extraction, genotyping and predictions

In this study, we selected polymorphisms of the following genes which are involved in angiogenesis process:

- VEGF-A (rs2010963G>C, rs699947A>C)
- VEGFR-2 (rs2305948C>T, rs1870377T>A)
- VEGFR-3 (rs307826T>C, rs307821C>A)

SNPs in the aforementioned genes were selected using National Center for Biotechnology Information (NCBI) data and reviewing medical literature, according to the following criteria:

- Polymorphisms were located in a biologically relevant area of the gene (i.e. intron, 5′ UTR and 3′ UTR or promoter region)
- minor allele frequency (MAF) was ≥ 10% (with the only exception of rs307821)
- genetic polymorphism was established and well documented.

Genomic DNA was extracted from whole blood using the *QIAamp DNA Mini QIAcube Kit*, according to the manufacturer’s procedures.

Polymorphisms genotyping was performed using pre-designed TaqMan SNP Genotyping Assays (Applied Biosystems, Foster City, CA), according to the manufacturer’s instructions. Amplifications and analysis were carried out on the 7300 Real-Time PCR System (Applied Biosystems), using the SDS software v1.4.0 for allelic discrimination (Applied Biosystems). About 10% of the samples were randomly remade for genotype confirmation and the results were 100% concordant. Data from general CEU population were provided by the HapMap project (http://www.HapMap.org). When these data were not available we considered the frequencies reported in the 1000 genome project (http://www.1000genomes.org).

### Statistical analysis

Disease Free Survival (DFS) was defined as the interval between the date of diagnosis to the date of disease progression or death or last follow-up visit in patients not yet relapsed. DFS distribution was estimated using the Kaplan-Meier method and Mantel-Haenszel log-rank test was employed to compare survival among groups. A Cox-regression model was applied to the data with a univariate approach and used to assess the role of polymorphisms as prognostic factors. Any variable having *p* < 0.20 at univariate analysis was selected as a candidate for the logistic regression analysis with a significance levels set at a 0.05 value [21, 22].

The genotype frequencies of VEGF-A, VEGFR2, VEGFR3, were checked for the Hardy–Weinberg equilibrium (HWE) and linkage disequilibrium (LD) using Haploview, (Broad Institute, Cambridge, MA) to ensure that the markers were appropriate for inclusion in the haplotype estimates. The LD was measured by the disequilibrium coefficient (D), and LD significance was considered at a D ≥ 80%. The most common genotypes in control subjects were considered as references. Association between categorical variables was checked by using a chi-square test and a Fisher’s exact probability test. The Benjamini-Hochberg correction method was used to adjust the values for multiple comparisons [23].

Statistical analysis was performed with MedCalc software version 11.4.4.0 (MedCalc Software, Br ockstreet 52, 9030 Mariakerke, Belgium).

## Results

Fifty-eight patients with histologically or cytologically proven diagnosis of GEP-NENs were evaluated in this study. Clinical and pathological characteristics are summarized in Table 1.

**Table 1:** Patients’ characteristics.

Parameters	Patients (N = 58)
**Gender**	
Male	32 (55.2%)
Female	26 (44.8%)
**Age at the diagnosis—yr**	
Median	57
Range	24–79
**Site of primary tumor**	
Pancreas	45 (77.5%)
Small intestine	6 (10.5%)
Large intestine	3 (5.0%)
Stomach	2 (3.0%)
Duodenum	1 (2.0%)
Appendix	1 (2.0%)
**Histological grading**	
G1	27 (46.5%)
G2	28 (48.3%)
G3	3 (5.2%)
**Stage at the diagnosis**	
I	9 (15.5%)
IIa	12 (21.0%)
IIb	4 (7.0%)
IIIa	3 (5.0%)
IIIb	8 (13.5%)
IV	22 (38.0%)
**Exitus**	
Yes	3 (5.2%)
No	55 (94.8%)

According to previous surgical and medical history (Table 2), 51 patients (86.4%) underwent surgical resection. Twenty-seven patients (46.6%) received a first-line treatment consisting in SSAs (44.8%), PRRT (25.9%), everolimus (12.1%), chemotherapy (10.3%) or other therapies (3.4%). After progression to first line therapy, 9 patients performed a second-line, 3 patients a third-line and only 1 patient a fourth-line therapy.

**Table 2:** Surgical and medical history of the enrolled patients.

Parameters	Patients (N = 58)
**Surgery**	
Not performed	7 (12.1%)
Performed	51 (87.9%)
• Radical surgery	40 (78.4%)
• Debulking and/or metastasectomy	11 (21.6%)
**First-line medical treatment**	
Not performed	31 (53.4%)
Performed	27 (46.6%)
• Somatostatin analogues	26 (44.8%)
• Peptide receptor radionuclide therapy	15 (25.9%)
• Everolimus	7 (12.1%)
• Chemotherapy	6 (10.3%)
• Other	2 (3.4%)
**Second-line medical treatment**	
Not performed	49 (84.5%)
Performed	9 (15.5%)
**Third-line medical treatment**	
Not performed	55 (94.8%)
Performed	3 (5.2%)
**Fourth-line medical treatment**	
Not performed	57 (98.3%)
Performed	1 (1.7%)

In our series, disease progression was observed in 43% of patients with a median PFS of 46.0 months (range 0.1 to 91.0 months).

At univariate analysis, patients with lower tumor burden (T3) had a longer PFS than those with larger tumors (T4) (46.0 months vs. 4.0; *p* = 0.0001). Furthermore, patients presenting stage IV at diagnosis had a significantly lower PFS than patients without metastasis at onset (5.4 months vs. 46.0 months, *p* = 0.0009). Finally, a trend towards a better PFS in females (49.2 months vs. 27.8 months; *p* = 0.405), and in patients older than 65 years compared to younger patients (61.9 months vs. 27.8 months, *p* = 0.258) was observed. At multivariate analysis, only tumor burden (referring to the size of tumor) resulted an independent prognostic factor (*p* = 0.0086).

### Analysis of polymorphisms

Two SNPs were identified respectively in VEGF-A (rs2010963, rs699947), VEGFR-2 (rs2305948, rs1870377), and VEGFR-3 (rs307821, rs307826) gene. Chromosomal location, position in the gene, effect and codon/aminoacid exchange are shown in Table 3.

**Table 3:** Chromosomal location, position in the gene, effect and codon/aminoacid exchange of polymorphism studied group.

SNP	Gene	Chromosome	Position/effect	Codon exchange	AA exchange
rs2010963	VEGF-A	6	5’-UTR	—	—
rs699947	VEGF-A	6	Promoter	—	—
rs1870377	VEGFR-2	4	Missense	CAA→CAT	Q[Gln]→H[His]
rs2305948	VEGFR-2	4	Missense	GTA→ATA	V[Val]→I[Ile]
rs307821	VEGFR-3	5	Missense	CGC→CAG	R[Arg]→Q[Gln]
rs307826	VEGFR-3	5	Missense	ACG→GCG	T[Thr]→A[Ala]

All SNPs were in HWE. The LD analysis revealed that VEGFA rs2010963 and rs69947 were in strong LD. The frequencies of SNPs in GEP-NENs have been compared with those in the general population (Table 4).

**Table 4:** Genotype and allele frequencies of evaluated SNPs.

GENE	SNPs	Allele	Frequencies general population	Frequencies Study cohort	n. sample
VEGFR 2	rs2305948	C	92.00%	87.93%	58/58
		T	8.00%	12.07%	
VEGFR 2	rs1870377	T	72.50%	71.55%	58/58
		A	27.50%	28.45%	
VEGF A	rs2010963	G	68.82%	65.52%	58/58
		C	31.18%	34.48%	
VEGF A	rs699947	C	52.20%	50.88%	57/57
		A	47.80%	49.12%	
VEGFR3	rs307821	C	90.59%	90.52%	58/58
		A	9.41%	9.48%	
VEGFR3	rs307826	T	89.80%	89.47%	57/57
		C	10.20%	10.53%	

VEGFR-2 rs2305948 T polymorphism frequency was higher in GEP-NENs than in the general population (12.07% vs. 8.00%), as well as VEGF-A rs2010963 C polymorphism (34.48% vs. 31.18%). The remaining allele frequencies are almost identical in the two populations.

We further investigated the prognostic role of SNPs on DFS.

Three out SNPs showed a correlation with an increased risk of disease relapse. The presence of VEGF-A rs2010963 GC genotype correlates with a lower DFS than the presence of homozygous GG (27.8 months vs. 49.2 months, *p* = 0.0504; HR: 0.4665) (Fig 1A). Furthermore, patients with VEGF-A rs699947 C and CA genotypes showed a trend towards a worse DFS than those with A (27.8 months vs. 61.9; *p* = 0.105; HR: 0.4832) (Fig 1B). A correlation between VEGFR-3 rs307821 C genotype and a lower DFS compared to A and CA was observed (46 months vs. 61.9 months; *p* = 0.2062) (Fig 1C).

**Fig 1:** Progression free survival (PFS, expressed in months) according to selected VEGF-A, VEGFR-2 and VEGFR-3 polymorphisms. a) VEGF-A polymorphisms. b) VEGFR-2 polymorphisms. c) VEGFR-3 polymorphisms. d) Poor group (patients presenting all 3 polymorphisms) vs not poor group (patients presenting 1 or 2 polymorphisms). e) High-risk group (patients presenting all 3 polymorphisms) vs intermediate-risk group (patients presenting 2 polymorphisms) vs low-risk group (patients presenting at most 1 polymorphisms).

According to the presence of all the genotypes with negative prognostic value (rs2010963 GC, rs699947 AC and C and rs307821 C), patients were stratified in two subpopulations identifying a group of 31 patients (53.4%) with unfavorable biological characteristics (*poor group*). Statistical analysis showed that the poor group has a significantly lower DFS compared to the remaining patients (27.8 months vs 49.2 months, *p* = 0.0141; HR: 0.3935) (Fig 1D). Finally, we grouped the patients according to the number of polymorphisms with negative prognostic value, detecting three different subgroups:

1. *Poor group or high-risk group*: represented by patients presenting all 3 polymorphisms with unfavorable prognostic significance;
2. *Intermediate-risk group*: patients presenting 2 polymorphisms with unfavorable prognostic significance;
3. *Low-risk Group*: patients presenting at most one of the polymorphisms with unfavorable prognostic significance.

The *high-risk group* include 31 patients (53.4%); 15 patients (25.9%) belong to the *intermediate-risk group*, while the remaining 12 patients (20.7%) are at *low-risk group*. A statistically significant difference in terms of DFS (*p* = 0.0342) was observed between these three different groups, with 61.9 months in the *low-risk group*, 49.2 months in the *intermediate-risk group* and 27.8 months in the *poor-risk group* (Fig 1E).

## Discussion

In our study, we aimed to analyze the prognostic and predictive role of angiogenic factors in GEP-NENs through the analysis of SNPs of angiogenic markers.

The following SNPs, VEGF-A rs699947C, VEGF-A rs2010963GC and VEGFR-3 rs307821C, significantly correlated with a shorter progression free survival (PFS) suggesting, for the first time, that abnormalities in VEGF pathway might act as prognostic factors in GEP-NENs.

Many studies have investigated the prognostic significance of angiogenesis’ SNPs in several tumors, including breast cancer [24], glioma [25], colorectal cancer [26], lung cancer [27], oral squamous cell carcinoma [28], renal cell carcinoma [29]. We have also previously shown their role in thymic malignancies [30]. However, a potential role in neoplasm susceptibly as well as the prognostic significance of SNPs in VEGF pathway have not been defined in neuroendocrine neoplasms, yet.

Our results showed an increased frequency of VEGFR-2 rs2305948T and VEGF-A rs2010963C polymorphisms in GEP-NEN than in general population, thus suggesting that these SNPs may represent peculiar risk factors for the occurrence of neuroendocrine tumors.

We also investigated the prognostic role of several SNPs in patients with GEP-NENs.

We found that VEGF-A rs2010963GC polymorphism correlated with lower PFS than homozygous GG (27.8 months vs. 49.2 months, *p* = 0.0504). This polymorphism has already been studied in other tumor types proving an association with an increased risk of developing glioma in Chinese population [31] and cervix intraepithelial neoplasia [32]. Bhaskari *et al*. showed also a correlation with the presence of ascites in an Indian ovarian cancer patients [33]. Furthermore, our group has previously demonstrated the predictive role of rs2010963 in patients with renal cell carcinoma treated with sunitinib [29] and has also confirmed this role in patients with hepatocellular carcinoma treated with sorafenib [34] and in metastatic colorectal cancer patients treated with regorafenib [35]. Thus proving that it is an independent factor for both progression-free survival and overall survival. In particular VEGF-A rs2010963CC polymorphism resulted linked to improved outcome both in HCC and mCRC while in our study VEGF-A rs2010963 GC genotype correlates with a lower DFS, maybe because GEP-NENs patients included in our study were totally antiangiogenic naïve.

Furthermore, in our study, the other VEGF-A polymorphism demonstrated a correlation with DFS: patients with VEGF-A rs699947C and CA genotypes showed a trend towards worse DFS than those with genotype A (27.8 months vs 61.9; *p* = 0.105; HR: 0.4832). In line with our results, VEGF-A rs699947A polymorphism seems to be associated with longer progression-free survival and overall survival in patients with renal cell carcinoma treated with sunitinib [29], whilst Masago *et al*. showed a positive prognostic role of VEGF-A rs699947C polymorphism in patients with non-small cell lung cancer [36]. Moreover, other studies focused on the role of this polymorphism in tumor susceptibility concluding that the rs699947C seems to have a protective effect against colorectal cancer [37].

In our study, we also observed a correlation between VEGFR-3 rs307821C genotype and DFS compared to A and CA (46 months vs 61.9 months; *p* = 0.2062) (Fig 1C). Literature data about rs307821 polymorphism are scarce, mostly focusing on other SNPs of the same gene. VEGFR-3 rs307821 polymorphism has been previously evaluated in patients with renal cell carcinoma treated with sunitinib showing a significant correlation with overall survival and disease free survival [38, 39]. Recently, rs307821 was studied in patients with neuroendocrine tumors treated with pazopanib within PAZONET trial proving to have a significant prognostic value [40].

Vascular endothelial growth factors (VEGFs) and their three structurally related receptors (VEGFRs) represent master regulators of vessels functions in physiological and pathological processes. Angiogenesis represents a key event in cancer development. VEGFR-2 is the main receptor involved in promoting angiogenesis through two main mechanisms, intussusception and sprouting [41]. In fact binding of VEGF-A to VEGFR-2 promotes proliferation of endothelial cells through activation of the RAS/RAF/ERK/ MAPK pathway [42, 43] and, at the same time, induces the expression of antiapoptotic protein prolonging their survival [44]. VEGFR-3 is the principal regulator of lymphendothelial cell proliferation, migration and apoptosis; nevertheless, this receptor is been found out also in endothelial cells and its expression becomes up-regulated during active angiogenesis as in tumor vasculature. Furthermore VEGF-A, C and D could induce heterodimerization of VEGFR-2 and VEGFR-3 activating signal transduction pathway involved in angiogenesis modulation [41].

On this basis, the abnormalities in VEGF pathway detected in GEP-NETs might promote angiogenesis process virtually increasing the aggressiveness of the disease.

To the best of our knowledge, the present study is the first to investigate the prognostic significance of SNPs of VEGF pathway in GEP-NENs. The results of our study suggest that SNPs analysis may be useful in order to identify high-risk group of GEP-NENs characterized by poor prognosis and more likely that could benefit from treatment with anti-angiogenic agents. Currently, sunitinib represents the only anti-angiogenic drug approved in Pan-NET, but other clinical trials are still ongoing, evaluating other agents of the same category. These results might allow to better stratify patients with GEP-NENs in order to offer a more personalized therapy.

However, we that our findings will require confirmation in perspective larger epidemiological studies focusing on the prognostic significance of SNPs in GEP-NENs helping clinicians to optimize the management of these heterogeneous tumors.

## Supporting information

S1 Dataset Minimal data set about patients included in our study. (XLSX)
